RETRACTED

# Early or delayed cord clamping during transition of term newborns: does it make any difference in cerebral tissue oxygenation?

**DOI:** 10.1186/s13052-024-01707-9

**Published:** 2024-07-29

**Authors:** Baran Cengiz Arcagok, Hulya Bilgen, Hulya Ozdemir, Asli Memisoglu, Dilsad Save, Eren Ozek

**Affiliations:** 1 Department of Pediatrics, Division of Neonatology, School of Medicine, Acibadem University, Istanbul, Turkey; 2 Department of Pediatrics, Division of Neonatology, School of Medicine, Marmara University, Istanbul, Turkey; 3 Department of Public Health, School of Medicine, Marmara University, Istanbul, Turkey

**Keywords:** Delayed cord clamping, Term newborn, Cerebral tissue oxygenation, Near-infrared spectroscopy, Fractional tissue oxygen extraction

## Abstract

**Background:**

According to the World Health Organization’s recommendation, delayed cord clamping in term newborns can have various benefits. Cochrane metaanalyses reported no differences for mortality and early neonatal morbidity although a limited number of studies investigated long-term neurodevelopmental outcomes. The aim of our study is to compare the postnatal cerebral tissue oxygenation values in babies with early versus delayed cord clamping born after elective cesarean section.

**Methods:**

In this study, a total of 80 term newborns delivered by elective cesarean section were included. Infants were randomly grouped as early (clamped within 15 s, n:40) and delayed cord clamping (at the 60th second, n:40) groups. Peripheral arterial oxygen saturation (SpO2) and heart rate were measured by pulse oximetry while regional oxygen saturation of the brain (rSO2) was measured with near-infrared spectrometer. Fractional tissue oxygen extraction (FTOE) was calculated for every minute between the 3rd and 15th minute after birth. (FTOE = pulse oximetry value-rSO2/pulse oximetry value). The measurements were compared for both groups.

**Results:**

The demographical characteristics, SpO2 levels (except postnatal 6th, 8th, and 14th minutes favoring DCC *p* < 0.05), heart rates and umbilical cord blood gas values were not significantly different between the groups (*p* > 0.05). rSO2 values were significantly higher while FTOE values were significantly lower for every minute between the 3rd and 15th minutes after birth in the delayed cord clamping group (*p* < 0.05).

**Conclusion:**

Our study revealed a significant increase in cerebral rsO2 values and a decrease in FTOE values in the delayed cord clamping (DCC) group, indicating a positive impact on cerebral oxygenation and hemodynamics. Furthermore, the DCC group exhibited a higher proportion of infants with cerebral rSO2 levels above the 90th percentile. This higher proportion, along with a lower of those with such parameter below the 10th percentile, suggest that DCC may lead to the targeted/optimal cerebral oxygenetaion of these babies. As a result, we recommend measuring cerebral oxygenation, in addition to peripheral SpO2, for infants experiencing perinatal hypoxia and receiving supplemental oxygen.

RETRACTED

## Background

Although clamping the umbilical cord at birth is the oldest intervention in humans, the optimal timing of cord clamping has been a subject of controversy for years [1–3]. Numerous randomized controlled trials have compared the benefits of early cord clamping (ECC) versus delayed cord clamping (DCC), which is generally defined as clamping the umbilical cord 60 s after birth. Based on these studies, more specific recommendations have been proposed regarding the optimal timing for umbilical cord clamping, especially for infants who are large for gestational age and with intrauterine growth restriction. [4–11].

Previous studies in term infants have shown that approximately 80 ml of blood, known as placental transfusion, is transferred from the placenta to the newborn one minute after birth, and this amount increases to approximately 100 ml three minutes after birth [12, 13]. Placental transfusion may improve circulating volume at birth, which, in turn, may improve outcomes in preterm infants [14–16]. Several systematic reviews have suggested that delaying umbilical cord clamping, with the infant maintaned at or below the level of the placenta, can yield various benefits. These benefits include higher hemoglobin and hematocrit levels during the early neonatal period [17–20], increased total body iron stores [19, 21], elevated circulating ferritin levels at 2–4 months of age [4, 21], and a lower incidence of iron deficiency anemia at around 4 months of age [12, 18, 22] in term infants.

The measurement of regional cerebral tissue oxygen saturation (rSO_2_) using near-infrared spectroscopy (NIRS) allows for noninvasive monitoring of brain oxygenation in both preterm and term infants [23]. This technique may provide information to help preventing brain damage during the transition from the fetal to the neonatal period [23–25]. Monitoring cerebral rSO_2_ enables to ensure that the baby is receiving adequate oxygen supply, which is essential for proper brain development and overall health [26, 27]. The aim of our study is to compare postnatal cerebral tissue oxygenation values in term infants with ECC versus DCC born after elective cesarean section (C/S).

## Materials and methods

### Study design and ethical approval

This prospective randomized study enrolled 80 term newborns delivered by elective cesarean section (C/S) between 37 + 0/7 weeks and 41 + 6/7 weeks from uncomplicated singleton pregnancies. Exclusion criteria included parental refusal to participate, major congenital anomalies, multiple pregnancies, placental abruption, uterine rupture, maternal use of medications affecting the fetus, and severe maternal illness or suspected/proven infection of the newborn. The newborns were categorized into two groups based on the timing of cord clamping: early clamping (within 15 s, *n* = 40) and delayed cord clamping (at the 60th second, *n* = 40). The research staff, prior to delivery, randomly allocated newborns into these groups by opening sequentially numbered opaque randomization envelopes. This study protocol was reviewed and approved by the Regional Committee on Biomedical Research Ethics. Written informed constent was obtained from the parents.

RETRACTED

### Monitoring procedures

Following birth, neonates were positioned between their mother’s thighs. Subsequent to cord clamping, a NIRS sensor was placed on the left forehead, and a pulse oximeter sensor was additionally secured on the right palm or wrist to monitor pre-ductal arterial oxygen saturation (SpO2) and heart rate (HR). Peripheral SpO2 and HR were measured by pulse oximetry (Covidien Nellcor N200, Minneapolis, USA), while cerebral rSO2 was measured by a near-infrared spectrometer with the neonatal transducer (Invos 5100 C, Medtronic, Minneapolis, MN). Total bilirubin was measured using a transcutaneous bilirubinometer (Draeger Jaundice Meter JM-103, Draeger Medical, Inc., Telford, PA, USA) at 24 h of postnatal age.

### Possible criticisms on sensor placement

The placement of the NIRS sensor may be subject to criticism, as the reliability of cerebral oxygenation measurements can be influenced by sensor positioning. We acknowledge this potential limitation and took utmost care to ensure consistent and accurate placement. However, variations in the precise location of the sensor could have affected the recorded data.

### Outcome measures

Measurements of SpO2, HR and cerebral rSO_2_ were recorded every minute between the 3 and 15 min after birth. FTOE was calculated for each minute (FTOE = pulse oximetry value-rSO2/pulse oximetry value). Hematocrit levels were measured at the postnatal 2nd hour, and bilirubin levels were measured at the postnatal 24th hour for all infants. Blood samples for blood gas analyses were collected from the umbilical arteries immediately after cord clamping. The measurements and analyses were compared between the early and delayed cord clamping groups. The primary outcome aimed to compare postnatal cerebral tissue oxygenation values in term infants with ECC versus DCC, while the secondary outcome involved the comparison of SpO2, HR, hematocrit, and bilirubin levels between the two groups.

RETRACTED

### Statistical analysis

Descriptive statistics were presented as mean and standard deviation (SD), or median and interquartile range (IQR) when the data follow nonparametric distribution. Baseline characteristics of early and delayed cord clamping groups were compared using independent samples T-test, or Mann-Whitney U test when parametric assumptions were violated, and Chi-square test for the categorical variables. The comparison between the groups over the study period was investigated with Repeated measure two-way ANOVA Greenhouse-Geisser. Statistical tests were two-tailed and conducted at 5% significance level. The statistical analysis was performed using SPSS for Windows version 19.0 (SPSS Inc, Chicago, Illinois, USA).

## Results

A total of 80 term newborns were enrolled in the study, with their median gestational weeks and birth weights categorized based on the type of cord clamping as follows: 38.50 (38–39) weeks in the ECC group, 39.00 (38–39) weeks in the DCC group, and 3355 (3080–3576) grams in the ECC group, 3400 (3125–3800) grams in the DCC group, respectively. The demographic characteristics, including gestational age, birth weight, and gender, were comparable between the two groups. The Apgar score at the fifth minute was significantly lower in ECC group than DCC group (*p* < 0.01), there was no statistically significant difference at the tenth minutes (*p* > 0.05). Detailed comparisons of demographic characteristics, Apgar scores, cord blood gas, and laboratory test results based on the type of cord clamping are presented in Table 1.

**Table 1:** Comparison of the demographic features and laboratory test results of the infants

Variable	Early cord clamping (*n* = 40)	Delayed cord clamping (*n* = 40)	*p*-value
Sex (female/male)¹	26/14	20/20	0.175^a^
Birthweigth (gr)²	3355.00 (3080.00–3576.25)	3400.00 (3125.00–3800.00)	0.799^b^
Gestational age (weeks)²	38.50 (38.00–39.00)	39.00 (38.00–39.00)	0.240^b^
Apgar scores_5 minute_²	10.00 (9.00–10.00)	10.00 (10.00–10.00)	0.007^b^*
Apgar scores_10 minute_²	10.00 (10.00–10.00)	10.00 (10.00–10.00)	0.050^b^
pH³	7.31 ± 0.04	7.32 ± 0.04	0.300^c^
pCO_2_ (mm/Hg)³	48.64 ± 5.82	47.67 ± 6.61	0.490^c^
HCO_3_ (mm/Hg)³	23.72 ± 1.91	23.75 ± 1.98	0.954^c^
Lactate (mmol/liter) ²	1.70 (1.40–2.32)	1.85 (1.50–2.52)	0.215^b^
Hematocrit³	56.25 ± 4.09	59.98 ± 3.41	< 0.001^c^*
Bilirubin²	2.35 (1.95–3.32)	3.40 (2.80–3.82)	< 0.001^b^*

Descriptives reported with ¹frequency, ²median (interquartile range), ³mean ± SD. *p*-values for ^a^Chi-square test, ^b^Mann-Whitney U test, and ^c^Independent samples T-test.*p-value < 0.05

RETRACTED

### Primary endpoint

The primary endpoint of this study was to evaluate the impact of cord clamping timing on cerebral rSO2 and FTOE.

### Secondary endpoints

Comparison of SpO2 and HR levels (Table 2; Fig. 1).

**Table 2:** Comparison of SpO_2_ and HR according to the type of cord clamping

	Early cord clamping (mean ± SD)	Delayed cord clamping (mean ± SD)	*p*-value^a^
SpO_2_ 3´	71.75 ± 12.093	72.38 ± 9.131	0.795
SpO_2_ 4´	75.55 ± 12.979	78.75 ± 8.418	0.195
SpO_2_ 5´	78.75 ± 12.957	82.93 ± 7.950	0.086
SpO_2_ 6´	81.28 ± 11.435	86.15 ± 6.800	0.023*
SpO_2_ 7´	84.90 ± 9.128	88.13 ± 5.992	0.066
SpO_2_ 8´	87.23 ± 7.911	89.65 ± 5.241	0.011*
SpO_2_ 9´	88.80 ± 7.318	91.25 ± 4.199	0.070
SpO_2_ 10´	90.08 ± 6.753	91.85 ± 4.555	0.172
SpO_2_ 11´	90.48 ± 5.542	92.05 ± 4.391	0.163
SpO_2_ 12´	90.43 ± 5.710	92.53 ± 4.391	0.069
SpO_2_ 13´	91.53 ± 4.772	92.95 ± 4.082	0.155
SpO_2_ 14´	91.75 ± 5.527	93.85 ± 3.641	0.048*
SpO_2_ 15´	92.30 ± 5.576	93.88 ± 3.531	0.135
HR 3´	162.88 ± 17.440	165.08 ± 13.746	0.533
HR 4´	162.38 ± 17.545	162.78 ± 12.612	0.907
HR 5´	164.25 ± 15.713	162.18 ± 11.899	0.507
HR 6´	162.05 ± 14.322	159.05 ± 11.377	0.303
HR 7´	159.55 ± 15.009	157.50 ± 12.886	0.514
HR 8´	158.68 ± 15.366	156.45 ± 13.095	0.488
HR 9´	156.88 ± 14.460	154.10 ± 12.717	0.365
HR 10´	155.85 ± 14.894	153.03 ± 10.807	0.335
HR 11´	155.25 ± 16.274	152.43 ± 12.553	0.387
HR 12´	151.78 ± 27.193	153.93 ± 11.881	0.648
HR 13´	155.78 ± 17.210	153.18 ± 11.871	0.434
HR 14´	154.23 ± 16.493	152.58 ± 11.931	0.610
HR 15´	153.78 ± 15.993	152.43 ± 11.993	0.670

^a^Independent samples T-test *p*-values comparing early (*n* = 40) and delayed (*n* = 40) cord clamping groups.*two-tailed *p*-value < 0.05

**Fig. 1:** Course of SpO_2_ and HR values according to the type of cord clamping

Assessment of umbilical cord blood gas values.

Assessment of bilirubin, hematocrit.

### Main findings

Other than the SpO_2_ levels at the 6th, 8th and 14th minutes (*p* < 0.05), HR, umbilical cord blood gas value and SpO_2_ levels did not show significant differences between the groups (*p* > 0.05) (Table 2).

The mean cerebral rSO2 levels were significantly higher, and the mean FTOE levels were significantly lower in the DCC group than the ECC group for each minute (*p* < 0.05) (Table 3).

**Table 3:** Comparison of cerebral rSO_2_ and FTOE according to the type of cord clamping

	Early cord clamping (mean ± SD)	Delayed cord clamping (mean ± SD)	*p*-value^a^*
rSO_2_ 3´	38.9 ± 23.228	54.15 ± 18.669	0.002
rSO_2_ 4´	46.33 ± 25.05	66.20 ± 17.067	< 0.001
rSO_2_ 5´	55.35 ± 25.617	74.83 ± 14.799	< 0.001
rSO_2_ 6´	62.53 ± 22.959	81.85 ± 11.672	< 0.001
rSO_2_ 7´	69.65 ± 19.232	86.05 ± 9.375	< 0.001
rSO_2_ 8´	73.13 ± 15.542	87.75 ± 8.006	< 0.001
rSO_2_ 9´	77.55 ± 12.698	89.35 ± 6.112	< 0.001
rSO_2_ 10´	79.43 ± 9.120	90.83 ± 4.701	< 0.001
rSO_2_ 11´	76.70 ± 18.470	89.55 ± 5.940	< 0.001
rSO_2_ 12´	81.28 ± 7.805	89.43 ± 5.606	< 0.001
rSO_2_ 13´	81 ± 7.435	89.30 ± 5.478	< 0.001
rSO_2_ 14´	80.40 ± 8.142	89.18 ± 5.434	< 0.001
rSO_2_ 15´	80.55 ± 8.391	89.95 ± 5.124	< 0.001
FTOE 3´	0.487 ± 0.240	0.267 ± 0.187	< 0.001
FTOE 4´	0.420 ± 0.243	0.169 ± 0.158	< 0.001
FTOE 5´	0.328 ± 0.239	0.102 ± 0.128	< 0.001
FTOE 6´	0.253 ± 0.205	0.052 ± 0.092	< 0.001
FTOE 7´	0.191 ± 0.182	0.024 ± 0.077	< 0.001
FTOE 8´	0.168 ± 0.137	0.020 ± 0.082	< 0.001
FTOE 9´	0.128 ± 0.117	0.020 ± 0.057	< 0.001
FTOE 10´	0.117 ± 0.082	0.009 ± 0.068	< 0.001
FTOE 11´	0.150 ± 0.201	0.025 ± 0.073	< 0.001
FTOE 12´	0.099 ± 0.085	0.032 ± 0.066	< 0.001
FTOE 13´	0.113 ± 0.087	0.038 ± 0.058	< 0.001
FTOE 14´	0.122 ± 0.085	0.048 ± 0.060	< 0.001
FTOE 15´	0.126 ± 0.087	0.040 ± 0.063	< 0.001

^a^Independent samples T-test *p*-values comparing early (*n* = 40) and delayed (*n* = 40) cord clamping groups.*two-tailed *p*-value < 0.05

The increase in cerebral rSO2 was faster, and the cerebral rSO2 plateau was reached earlier in the DCC group (Fig. 2).

RETRACTED

**Fig. 2:** Course of rSO2 and FTOE values according to the type of cord clamping

The number of infants with cerebral rSO2 levels above the 90th percentile was higher in the DCC group.

Bilirubin and hematocrit levels were also statistically higher in DCC group than ECC group (*p* < 0.05) without the need for phototherapy. Although the evaluation of bilirubin levels at 24 h may be early, no admission for phototherapy or other interventions has been observed in the DCC group.

The comparison of SpO_2_, HR, cerebral rSO_2_ and FTOE levels according to the type of cord clamping over the study period is shown in Table 4. The SpO2 level measured during the study progressively increased (*p* < 0.001), and this change in increase was similar between the groups (*p* > 0.05). The HR decreased during the study period (*p* < 0.001), and this change in decrease was similar between the groups (*p* > 0.05). The level of rSO_2_ was elevated over time (*p* < 0.001), and the change was significantly higher in DCC group than the ECC group (*p* < 0.001). The level of FTOE declined significantly throughout the study period between the study groups (*p* < 0.01). The decrease in FTOE level was higher in ECC group than DCC group (*p* < 0.001).

**Table 4:** Comparison of SpO_2_, HR, cerebral rSO_2_ and FTOE according to the type of cord clamping over the study period

Variable	Main Effect (F; *p*; $\:{\eta\:}^{2}$)^a^		Interaction effect (F; *p*; $\:{\eta\:}^{2}$)^a^
	Time	Group	Time x Group
SpO_2¹_	F = 162.37; *p* < 0.001; $\:{\eta\:}^{2}=$0.421*	F = 3.30; *p* = 0.073; $\:{\eta\:}^{2}=$0.015	F = 1.27; *p* = 0.286; $\:{\eta\:}^{2}=$0.003
HR	F = 20.15; *p* < 0.001; $\:{\eta\:}^{2}=$0.067*	F = 0.258; *p* = 0.613; $\:{\eta\:}^{2}=$0.002	F = 0.99; *p* = 0.412; $\:{\eta\:}^{2}=$0.003
rSO_2_	F = 100.11; *p* < 0.001; $\:{\eta\:}^{2}=$0.380*	F = 46.00; *p* < 0.001; $\:{\eta\:}^{2}=$0.116*	F = 2.91; *p* = 0.061; $\:{\eta\:}^{2}=$0.011
FTOE	F = 57.35; *p* < 0.001; $\:{\eta\:}^{2}=$0.272*	F = 66.70; *p* < 0.001; $\:{\eta\:}^{2}=$0.152*	F = 6.02; *p* = 0.003; $\:{\eta\:}^{2}=$0.029*

^a^Repeated measures two-way ANOVA Greenhouse-Geisser *p < 0.05 level

None of the infants were admitted to the Neonatal Intensive Care Unit.

RETRACTED

In summary, delayed cord clamping was associated with improved cerebral oxygenation, lower FTOE values, and favorable hematological outcomes compared to early cord clamping, highlighting the potential benefits of delayed cord clamping in term newborns.

## Discussion

Delayed cord clamping has been associated with positive outcomes in many studies. Beneficial effects such as higher hematocrit levels, lower anemia, and increased oxygenation have been observed [17–20, 28]. However, there is still a limited number of adequate studies in this field, and further research is needed. This article emphasizes the uncertainties surrounding the optimal timing of umbilical cord clamping. In our study, employing NIRS to measure cerebral rSO2, we sought to delve into the impact of DCC versus ECC in term infants born through elective cesarean section. The results show a significant advantage for the DCC group, with consistently higher cerebral rSO2 values and lower FTOE values, indicative of favorable cerebral oxygenation and hemodynamics. Notably, the DCC group exhibited a faster increase in cerebral rSO2, reaching a plateau earlier compared to the ECC group. The prevalence of infants with cerebral rSO2 levels above the 90th percentile was higher in the DCC group, underscoring the potential neuroprotective effects associated with delayed cord clamping. While these results particularly emphasize the importance of paying attention to the timing of cord clamping, especially in infants experiencing intrauterine hypoxia or requiring resuscitation [29, 30], it should be kept in mind that the prompt initiation of resuscitation maneuvers may be crucial for these infants.

A brief delay in clamping the umbilical cord following birth can impact cord blood gas values and potentially result in alterations in the acid-base balance [31]. In the randomized controlled studies various results have been reported. In the study by De Paco et al., and Anderson et al., no differences were found in the comparison of pH, pCO₂, lactate, HCO₃, and base deficit in the cord blood gas analysis. However, the pO₂ value was significantly higher in the DCC group [32, 33]. On the other hand in the study by Valero et al., and Wiberg et al., it was found that in the DCC group, pH, HCO_3_, base deficit, SaO₂ values were lower, while lactate values were higher [31, 34]. In another study conducted by Tanriverdi et al., no differences were observed in the blood gas parameters between the DCC and ECC groups [35]. In our study, we also did not find any significant differences in cord blood gas analyses, similar to the study conducted by Tanrıverdi et al., between the DCC and ECC groups. Our findings indicate that delaying cord clamping may not cause postnatal acidosis in infants.

RETRACTED

Several systematic reviews have suggested that clamping the umbilical cord in all births should be delayed for at least 30–60 s, with the infant maintaned at or below the level of the placenta because of the associated benefits [18–21]. Although there is a theoretical risk of symptomatic polycythemia and hyperbilirubinemia associated with placental transfusion, neither of these risks has been shown to be significant in current RCTs and observational studies [36–40]. Similarly, other studies have also reported significantly higher hematocrit levels in both preterm and term neonates in the DCC group compared with ECC group [6, 41–43]. In contrast to other studies, an observational study conducted by Consonni et al., did not find any difference in hematocrit levels at 48 h after birth between the groups [44].

The most feared side effect of delayed cord clamping is an increase in bilirubin levels due to elevated hemoglobin levels and the potential risk of Rh incompatibility and subsequent hemolytic newborn disease. Yang et al. found no significant difference in the mean peak serum bilirubin levels between ECC and DCC groups [36]. Studies that compared ECC and DCC in term newborns within the first 24 h, varying the duration from 30 s to 5 min or until cord pulsation ceased, found no variations in transcutaneous bilirubin levels [37–40]. The bilirubin levels and the need for phototherapy showed no significant differences between the groups [36, 39, 41]. According to the Cochrane review, infants who underwent DCC had higher hematocrit and bilirubin levels than infants who underwent ECC. However, these infants did not require any interventions or phototherapy [45]. In our study, hematocrit and bilirubin levels were found to be statistically higher in the DCC group compared to the ECC group (*p* < 0.05) without increasing the need for phototherapy or any intervention.

RETRACTED

SpO_2_ levels and HR of newborn infants during immediate transition are affected by the cord clamping time. In the study conducted by Cavallin et al., it was suggested that DCC is associated with a lower HR compared to ECC during the immediate postnatal phase, although this was close to statistical significance. In this study, oxygenation did not show any difference between the two clamping methods [6]. A different study that compared SpO_2_ and HR according to reference ranges provided by Dawson et al. (which were established when ECC was the standard of care), in early and delayed cord clamping groups, in healthy term infants delivered vaginally, found higher SpO_2_, lower HR values, and a lower HR increase during the initial minutes after birth, in the DCC group [46, 47]. This finding was not supported by another study in infants born via caesarean section, as no differences in SpO_2_ and HR were observed during the first 10 min after birth [48]. Similarly, we did not find any significant difference in HR and SpO_2_ levels during the immediate postnatal period between the groups. Moreover, a statistically significant difference favoring DCC was detected in SpO2 values at the postnatal 6th, 8th, and 14th minutes. These results show that neonates subjected to DCC do not experience any disadvantage in terms of cardiovascular adaptation and oxygenation compared to those undergoing ECC.

As a result of placental transfusion, tissue and organ perfusion are optimized simultaneously. Placental transfusion can also reduce the risk of hypoxic-ischemic brain injury in infants by affecting brain perfusion. Many studies, especially focusing on premature infants, have measured changes in brain oxygenation during the transition period after birth [49–53]. According to these studies, DCC improved cerebral oxygenation in such newborns [28, 53]. When examining the limited number of studies in the literature that measure brain tissue oxygenation in term infants during the transition period, we found very limited and not comprehensive data regarding the relationship between the duration of cord clamping and changes in cerebral hemodynamics [54–56]. In the literature, only two studies have investigated the relationship between cord clamping duration and brain oxygenation [57, 58]. In both studies, no statistically significant difference was found between the cord clamping time and cerebral tissue oxygenation. In our study we demonstrated that cerebral rsO_2_ values were significantly higher, while FTOE values were significantly lower in the DCC group compared to the ECC group between the 3 and 15 min after birth. Additionally the number of infants with cerebral rSO_2_ levels above the 90_th_ percentile was higher in the DCC group, while that of those with rSO2 below the 10th percentile was lower. The higher number of infants with rSO2 levels above the 90th percentile as a result of DCC actually indicates that the cerebral oxygenation of these babies is better. These findings emphasize the beneficial effect of DCC on cerebral oxygenation and cerebral hemodynamics.

RETRACTED

Although a number of randomized controlled trials in term and preterm infants have compared the benefits of DCC versus ECC, the ideal timing of cord clamping in specific situations remains unclear and requires further investigation. For example, infants requiring resuscitation may benefit significantly from placental infusion, but their need for immediate attention raises the question of whether cord clamping should be immediate or delayed. Therefore, in infants experiencing perinatal hypoxia and receiving supplemental oxygen, the measurement of cerebral oxygenation in addition to peripheral SpO2 might be considered.

While our study provides valuable insights into the effects of cord clamping timing on cerebral tissue oxygenation in term newborns, certain limitations should be acknowledged. First, the sample size in our study was relatively small, and the findings may benefit from validation in larger cohorts to enhance generalizability. Additionally, the study focused on newborns delivered by elective cesarean section, and extrapolating the results to infants delivered by other methods warrants caution. Furthermore, our analysis primarily concentrated on short-term outcomes, and the long-term neurodevelopmental implications of delayed cord clamping remain an area requiring further exploration. It is essential for future studies to include extended follow-up periods and comprehensive assessments to better elucidate the potential impact on cognitive and motor development.

## Conclusion

Our investigation aimed to assess the postnatal cerebral tissue oxygenation in term newborns subjected to early versus delayed cord clamping following elective cesarean section. Despite no significant differences found in demographic characteristics, SpO2 levels (except a few values), heart rates, and umbilical cord blood gas values between the groups, the number of infants with cerebral rSO2 levels above the 90th centile was higher in the DCC group. Based on these findings, we recommend the inclusion of cerebral oxygenation measurements, alongside peripheral SpO2, especially for newborns experiencing perinatal hypoxia and receiving supplemental oxygen. Additionally, our study emphasizes the utility of reference ranges and percentile charts for interpreting cerebral oxygenation during the immediate transition [59]. Integrating cerebral rSO2 reference ranges and percentile charts into monitoring during the fetal-to-neonatal transition holds promise in preventing adverse oxygenation outcomes during resuscitation.

RETRACTED

## Data Availability

The datasets used and/or analysed during the current study are available from the corresponding author on reasonable request.

## Abbreviations

ECC: Early cord clamping
DCC: Delayed cord clamping
rSO_2_: Regional cerebral tissue oxygen saturation
NIRS: Near-infrared spectroscopy
C/S: Cesarean section
SpO_2_: Oxygen saturation
HR: Heart rate
FTOE: Fractional tissue oxygen extraction
SD: Standart deviation
